# The Early Diagnostic Efficacy of Serum Histone H3 in Rabbit Urosepsis Model

This article has been retracted.

**DOI:** 10.1155/2021/9969344

**Published:** 2021-07-16

**Authors:** Xiaolu Zhang, Xiangcheng Zhan, Bisheng Huang, Saiyang Li, Yunfei Xu

**Affiliations:** ^1^Department of Urology, Shanghai Tenth People's Hospital, Tongji University School of Medicine, Shanghai 200072, China; ^2^Department of Urology, Changhai Hospital Affiliated to the Second Military Medical University/Naval Medical University, Shanghai 200433, China; ^3^Department of Urology, The Third Affiliated Hospital of Soochow University, Jiangsu 213003, China

## Abstract

**Objective:**

We want to explore the changing law of circulating histones in the acute stage of urosepsis and to find more sensitive and specific biomarkers for diagnosing urosepsis as early as possible.

**Methods:**

Twenty healthy male New Zealand rabbits were randomly divided into 4 groups (*N* = 5): the control group, sham group, model group of LPS 600 *μ*g/kg, and model group of LPS 1000 *μ*g/kg. Heart rate (HR), respiration rate (RR), rectal temperature (T), and mean arterial pressure (MAP) were examined at 1, 3, 6, 12, and 24 hours after operation. Besides, peripheral blood cell counts (RBC, WBC, PLT, and Hb) and C reaction protein (CRP) were tested at 1, 3, and 6 hours after operation, while the levels of histone H3, MMP-9, TIMP-1, and procalcitonin (PCT) in the serum were tested at 1, 3, and 6 hours after operation by ELISA. The heart, left lung, liver, and left kidney were harvested for HE stain and observed to research the pathological change of these tissues.

**Results:**

(1) The general status of rabbits: rabbits in the control and sham groups came out in 2 h after operation and regain to drink and eat in 12-24 h after operation. State of the rabbits in the control group was better than that in the sham group. Rabbits in the model groups were languid after operation and stopped to drink and eat. (2) Vital signs of rabbits: there was no statistic difference in HR (*P* = 0.238) and RR (*P* = 0.813) among all groups. MAP of the model groups decreased at 3 h postoperative, but transient (*P* < 0.001). The T of the LPS 1000 group decreased at 6 h postoperative (*P* = 0.003). (3) The change of biomarkers: H3 level of the LPS groups in the serum increased at 1 h postoperative (*P* < 0.01); MMP-9 of the LPS 1000 group increased at 1 h postoperative (*P* < 0.01); WBC of the model groups decreased at 3 h postoperative (*P* < 0.05); PLT of the LPS 1000 group is significantly increased at 1 h postoperative (*P* < 0.05); no statistic difference was found in CRP, PCT, and TIMP-1 among all groups. (4) Pathological sections: no abnormal performance was found in the control and sham groups. Glomerulus of the model groups was out of shape and necrosis with obvious renal tubule expansion. Pulmonary pathology showed alveolar septum diffuse increased and inflammatory infiltrate. Change of the LPS 1000 group was more serious than that of the LPS 600 group.

**Conclusions:**

Ligating the ureter after an injection of 1000 *μ*g/kg LPS into the ureter of the rabbit can establish the animal model of urosepsis. Histone H3 increase immediately at 1 h postoperative and are promised to be biomarkers of urosepsis, which are more effective than WBC, CRP, and PCT.

## 1. Introduction

Urinary stone disease (USD) is a common disease of urology with 1-5% morbidity while still on the rise in recent years. With the development of endoscopic urology, the main treatment of USD has changed from open operation to intracavitary lithotripsy [1]. At the same time, the incidence of postoperative complications has increased, including urosepsis. Urosepsis refers to sepsis caused by urinary tract or male reproductive organ infection, which accounts for about 5% of all sepsis. Previous reports indicated low incidence of urosepsis while the incidence of systemic inflammatory response syndrome (SIRS) and severe septic shock can be as high as 11.2-22% and 0.3-4.7% after intracavitary lithotripsy [2–6]. Moreover, asymptomatic urinary tract infections can be rapidly progressing to urosepsis in a short period of time; the mortality of the patients reaches 20-63%, which is a serious threat to the life and health of the patients. Although strengthening aseptic operation standard, shortening operation time, and placing ureteral stent can reduce the occurrence of postoperative infection, some high-risk factors such as complex stone, solitary kidney, and immune dysfunction cannot be avoided; urosepsis is still a difficult clinical problem to be solved.

Kumar et al. have shown that when sepsis occurs, the survival rate of the patients decreased by 8% per hour without sensitive antibiotics, and it is recommended to complete the bacterial culture and use of antibiotics within 1 h of onset [7]. According to the current diagnostic criteria, both infection evidence and signs of organ failure are needed, missing the window of early treatment [8–11]. Therefore, finding sensitive biomarkers in the early stage of sepsis is an effective way to improve the survival rate of the patient.

Histones are basic structural components of chromatin. The circulating histone in human body mainly comes from the passive release of dead or apoptotic cells and the active secretion of activated inflammatory cells [12]. Normally, histones released by chromatin collapse of dead cells are quickly cleared by monocytes, but in pathology cases, chromatin in the blood exceeds the metabolic capacity of the body; circulating histone level increases significantly [13–16]. Meanwhile, at the time of pathogen invasion, histone is secreted actively by activated inflammatory cells as neutrophil extracellular traps (NETs) and participates in the inflammatory response [17–19]. Among the five subtypes of histone, H3 and H4 are proved to be associated with this process [13].

H3 combines Toll-like receptor-2 (TLR2) and Toll-like receptor-4 (TLR4), taking part in various physiological and pathological processes [20]. In the previous study, Xu et al. demonstrated that H3 can directly damage endothelial cells and activate inflammatory signal pathway, promoting the release of cytokines such as tumor necrosis factor (TNF), leukocyte mediator (IL), and tissue factor (TF). In patients with sepsis, the median level of circulating H3 in the death group is significantly higher than that in the survival group; detecting nucleosome levels in the peripheral circulation helps evaluate the patients' prognosis [13]. In mouse sepsis model established by cecum puncture and ligation, histone antagonist reduces the damage of cardiac function [21]. Other researches also show that neutralizing H3 can improve the survival rate of sepsis mice [22], which prove that H3 plays an important role in the development of sepsis.

Sepsis model is commonly established by cecum puncture and ligation, or intra-abdominal injection of lipopolysaccharide (LPS) solution. However, the method of constructing uremic sepsis model is not clear [23]. In this study, we established the rabbit urosepsis model by ligating the ureter after injecting different concentrations of LPS solution into the ureter. Serum H3 level is detected compared with traditional diagnostic indexes of urosepsis such as PCT, CRP, and blood routine examination, so as to explore the sensitive and effective biomarkers for the early diagnosis of urosepsis.

## 2. Material and Methods

### 2.1. Material and Supplies

20 healthy male New Zealand rabbits provided from central laboratory of Shanghai Tenth People's Hospital were used. 4% paraformaldehyde solution was provided by central laboratory of Shanghai Tenth People's Hospital. Lipopolysaccharide (LPS, Sigma L6386-100MG), sodium heparin (Sigma H3149-500KU-9), chloral hydrate, xylazine hydrochloride injection, and the rabbit histone H3, matrix metalloproteinases-9 (MMP-9), procalcitonin (PCT), and tissue inhibitor of metalloproteinase-1 (TIMP-1) enzyme-linked immunosorbent assay (ELISA) kits were purchased commercially.

In animal model, rabbits were 2-3 months old and weighed between 1.61 and 3.30 (2.54 ± 0.45) kg. 20 rabbits were randomly assigned into the control group, sham group, experimental group of LPS 600 *μ*g/kg (LPS 600 group), and experimental group of LPS 1000 *μ*g/kg (LPS 1000 group). Each group had 5 rabbits. All rabbits were anesthetized using xylazine hydrochloride intramuscular injection at 1 mg/kg and 10% chloral hydrate intraperitoneal injection at 3 mL/kg. The distal segment of femoral artery was ligated, and the proximal segment was cannulated for measuring blood pressure and collecting blood. For rabbits of the sham group, the left ureter was identified and abdominal cavity was washed using 5 mL normal saline. For rabbits of the experimental groups, the distal segment of the left ureter was ligated and the proximal segment was cannulated and injected LPS solution. All the survived animals were sacrificed at 24 h after surgery.

### 2.2. Sample Collection and Measure

Cardiac rate, respiratory rate, and rectal temperature were measured at immediately, 1 h, 3 h, 6 h, 12 h, and 24 h after surgery. Blood samples were obtained at 1 h, 3 h, and 6 h after surgery. Fresh samples were used for routine blood and CRP test. Others were preserved at 4°C and centrifuged at 3000 rpm for 10 min. Supernatants were preserved at -80°C and used to test histone H3, MMP-9, TIMP-1, and PCT using enzyme-linked immunosorbent assay kit. Organization of the cardiac, lung, liver, and left kidney was obtained for pathological examination.

### 2.3. Statistical Analysis

One-way ANOVA test was used for comparison among all the groups. LSD test and Dunnett *t*-test were both used and take the major *P* value to compare the intergroup difference. *P* value < 0.05 was considered statistically significant. ROC curves were made using data of 1 h, 3 h, and 6 h to evaluate the predicting value of each parameter. IBM SPSS Statistics 25 software was employed for the analysis.

## 3. Results

### 3.1. Postoperation Reactions of Rabbits

#### 3.1.1. Control Group

All 5 rabbits wake up in 2 h after the operation and begin to eat and drink within 12 h. The form of excrement is normal, is sensitive to stimulations, quickly escapes from capture, and no mouth and nasal discharge were found. All rabbits are alive after 24 h.

#### 3.1.2. Sham Operation Group

All 5 rabbits wake up in 2 h and begin to eat within 12 h but the food intake is slightly less than that of the control. The form of excrement is normal, is sensitive to stimulations, capture is evasive, is slightly duller than the control group, and no eyes and nasal discharge were found. All rabbits survived 24 h after the operation.

#### 3.1.3. LPS 600 *μ*g/kg Group

We find that postoperative rabbits are somnolent, stop eating, slightly escape, and struggle when captured. They all have conjunctival congestion, with a small amount of yellow secretion in the mouth and nose. One rabbit dies 24 h after the operation, and the remaining 4 survived. The survived rabbits gradually return to autonomous gesture, and the conjunctival congestion recedes.

#### 3.1.4. LPS 1000 *μ*g/kg Group

One rabbit dies 3 h after the operation; others survive but are all in coma for the next 24 h, accompanied with severe conjunctival congestion and more mouth and nasal secretions. Two surviving rabbits are found with thrombosis in arterial catheterization.

### 3.2. Changes of Vital Signs of Rabbits

#### 3.2.1. Postoperation

There is no significant difference in heart rate, respiratory rate, and mean arterial pressure (MAP) among the groups (Figure 1). The anal temperature in the control group is 1°C higher than that in the rest groups (*P* = 0.007) (Figure 2). However, there is no difference in the postoperative groups indicating that the rise of the anal temperature is due to the operation (Table 1).

#### 3.2.2. 1 h after Operation

There is no significant difference in heart rate, respiratory rate, anal temperature, and MAP among the groups (Table 2).

#### 3.2.3. 3h after Operation

There is no significant difference in heart rate and respiratory rate among the groups. The anal temperature in the sham group is lower than that in the control group (*P* = 0.002), but no significant difference was found among the LPS group and sham group. MAP in both the experimental groups was lower than that in the sham group, and no significant difference was found between the sham and control groups (Table 3).

#### 3.2.4. 6 h after Operation

Anal temperature of the LPS 1000 group is lower than that in the sham group. There is no significant difference between the LPS 600 and sham groups because the results of LSD test (*P* = 0.018) and Dunnett *t*-test (*P* = 0.052) disagree. No difference was found in other parameters (Table 4).

#### 3.2.5. 12 h after Operation

Anal temperature in two experimental groups was lower than that in the sham group. No difference was found in other parameters (Table 5).

#### 3.2.6. 24 h after Operation

No difference was found in all parameters (Table 6).

### 3.3. Changes of Blood Routine and CRP

Platelet count 1 h after operation in the LPS 1000 group is (685.80 ± 150.52)∗10^9^/L, which is higher than (180.00 ± 70.06)∗10^9^/L in the sham group. And the increase of platelet continued to 6 h (Tables 7–9). But no similar change was found in the LPS 600 group. Leukocyte count 3 h after operation of the LPS 600 and LPS 1000 group is (3.86 ± 4.74)∗10^9^/L and (1.74 ± 0.40)∗10^9^/L, respectively, and both were significantly lower than that of the sham group (Table 8). Leukocyte count in the LPS 600 group at 6 h increased to (4.76 ± 4.06)∗10^9^/L, and that in LPS 1000 increased to (2.83 ± 0.96)∗10^9^/L (Figure 3). Both were lower than the sham group (Table 9). No significant difference was found in neutrophil count, erythrocyte, hemoglobin, and CRP (Tables 7–9).

### 3.4. Changes of Serum Histone, PCT, MMP-9, and TIMP-1

Concentration of histone H3 and H4 of the LPS 600 group at 1 h after operation was 5.71 ± 0.32 ng/mL and 2.89 ± 0.30 ng/mL, respectively. Histone H3 and H4 of the LPS 1000 group at 1 h after operation were 6.22 ± 0.57 ng/mL and 3.32 ± 0.26 ng/mL, respectively. All those parameters were significantly increased at 1 h after operation and stay to 6 h (Tables 10 and 11). Concentration of MMP-9 of the LPS 1000 group at 1 h after operation was 120.18 ± 18.46 ng/mL, which was significantly higher than the sham group (Table 12). Higher concentration of MMP-9 stayed to 3 h (136.10 ± 41.61 ng/mL) and 6 h (111.55 ± 12.21 ng/mL) after operation (Tables 10 and 11). For concentration of MMP-9, no similar change was found in the LPS 600 group. The change of concentration of PCT and TIMP-1 in the experimental groups had no statistical significance.

### 3.5. Comparison of Diagnostic Capability of Parameters

#### 3.5.1. Early Diagnostic

Serum histone H3/H4 and blood platelet count are earliest rising indicators among postoperative parameters (Figures 4–6). However, for MMP-9 and platelet count, only in the LPS 1000 group had statistical significance, which may mean these parameters just change in severe sepsis. At 3 h postoperation, MAP and leukocyte count significantly decreased, and concentration of H3, H4, MMP-9, and platelet count significantly increased. Similarly, only MMP-9 and platelet in the LPS 1000 group had statistical significance. MAP at 6 h postoperation increased to normal level; this could mean the change of blood pressure was transient so it could not be used for diagnosis. No significant difference was found in other parameters including heart rate, respiratory rate, CRP, PCT, and TIMP-1, so these parameters have no early diagnosis value.

#### 3.5.2. Sensibility and Specificity

The order of area under the curve (AUC) at 1 h postoperation was H3 (1.000) > H4 (0.970) > platelet count (0.950) > MMP − 9 (0.680). All these parameters had a diagnosis value except MMP-9 (*P* = 0.174 > 0.05), and the diagnosis value of H3 and H4 was better than others. The sensibility and specificity of H3 were both 100% when the cut-off is 5.04 ng/mL. The sensibility and specificity of H4 were 100% and 90%, respectively, when the cut-off is 2.62 ng/mL (Table 13, Figure 7).

The order of AUC at 3 h postoperation was H3 (1.000) = H4 (1.000) > platelet count (0.920) = leukocyte count (0.920) > MMP − 9 (0.710). MAP of experimental decreased transiently at 3 h postoperation so it has no diagnosis value. The sensibility and specificity of H3 and H4 were both 100% when the cut-off was 5.27 ng/mL and 2.87 ng/mL, respectively (Table 14, Figure 8).

The order of AUC at 6 h postoperation was H3 (1.000) = H4 (1.000) > leukocyte count (0.867) > platelet count (0.856) > MMP − 9 (0.822). All these parameters are diagnostic efficient and histone H3 and H4 have more advantages in specificity and sensitivity (Table 15, Figure 9).

### 3.6. Pathology at 24 h Postoperation

In the control group, no necrosis, hemorrhage, or inflammatory infiltration was observed in myocardial cells (Figure 10). Structure of alveoli was clear (Figure 11). Several minor bleeders were observed in pulmonary tissue. Structure of liver lobule and glomerulus was clear (Figure 12). What we observed in the sham group was similar to the control group. In the experimental groups, we observed karyopyknosis and breakage of the cardiomyocyte nucleus. We found necrosis of myocardial cells and inflammatory infiltration and hemorrhage in necrosis sections. No normal alveoli structure was observed in the experimental groups. And widespread bleeding and inflammation infiltration was found in the alveoli. Most liver cells in the experimental groups were edema and ballooning degeneration, and local inflammation was observed. Widespread renal tubular epithelial cell necrosis and glomerulus were severely out of shape (Figure 13). Casts were observed in enlarged lumen. All the changes above were more obvious in the LPS 1000 group.

## 4. Discussion

Millions of people suffer from sepsis worldwide every year, and the mortality rate can exceed 25%, which seriously threatens the life and health of human beings [9, 10]. Urosepsis accounts for about 5% of all sepsis, which is an important cause of death in urology patients, especially after urolithiasis surgery. The early diagnosis and treatment of sepsis have always been a vital but difficult point in the field of medicine. At present, two conditions should be met for the diagnosis of sepsis at the same time: (1) evidence of infection and (2) sequential organ failure score (SOFA) ≥ 2. The SOFA score included objective criteria for respiratory failure, coagulation dysfunction, elevated bilirubin, decreased blood pressure, disturbance of consciousness, and renal failure, lacking effective biomarkers for early diagnosis.

To explore the mechanism of the urosepsis occurrence and development, rational animal model is needed. Five kinds of modeling method are commonly used: (1) intravenous injection of exogenous toxin (commonly used LPS); (2) intravenous injection of bacterial suspension; (3) destruction of biological protection barrier of experimental animals; (4) manufacture of local soft tissue infection; and (5) pneumonia, meningitis model, etc. The method of constructing urosepsis remains unclear [21]. Patients undergoing intracavitary lithotripsy are susceptible to postoperative urinary sepsis and are now considered to be related to the interaction between the obstruction caused by urinary calculi and the infection [24]. In urinary tract obstruction combined with a sharp increase in intrarenal pressure during intracavitary lithotripsy, the toxin retrogrades into the blood circulation and eventually develops into urosepsis [25, 26]. We intend to simulate the nosogenesis by injecting the LPS solution into the ureter to induce urinary tract infection and ligating ureter to make ureteral obstruction. Given the difficulty of operation and postoperative evaluation, we selected New Zealand rabbits aged 2-3 months.

According to previous study, two LPS concentration gradients were set up in the experimental group, which were 600 *μ*g/kg and 1000 *μ*g/kg, respectively, in order to find out the suitable concentration of the model and simulate the different severity of infection. Histological and pathological examination was performed 24 hours after operation to confirm the establishment of the model. We set up the sham-operation group to exclude the influence of the operation on the result. All rabbits in the control group and sham operation group survive after the operation. Except for the transient hypothermia at a 3-hour postoperative time in the sham operation group (considering to be surgical factors), no infection-related clinical symptoms and signs are detected. Pathological results showed that the morphology of the heart, lung, liver, and kidney is basically normal, which proved that the operation itself would not cause urosepsis. On the contrary, in the LPS-treated groups, diffuse thickening of alveolar septum, massive infiltration of inflammatory cells in the alveoli, destruction of nephron, and disintegration of glomerular structure are found, indicating multiple organ failures of the rabbits; urosepsis model is successfully established. Thus, ligating the ureter after injection of LPS solution into the ureter can trigger urosepsis in rabbits.

Comparing the experimental group with the sham operation group, there is no significant change in postoperative heart and respiratory rate; anal temperature decreases significantly after 6 hours; mean arterial pressure returned to normal after a transient decrease at 3 hours after operation and remained at normal level until 24 hours. Therefore, the urosepsis cannot be diagnosed with these clinical indexes, but pathology confirms that the rabbits in the experimental groups have entered the early stage of sepsis. Peripheral blood WBC count (3.86 ± 4.74) × 10^9^/L in the LPS 600 group and (1.74 ± 0.40) × 10^9^/L in the LPS 1000 group is significantly lower than that in the sham group (9.84 ± 3.86) × 10^9^/L 3 hours after the operation. When it comes to 6 hours after the operation, the WBC count rises up to (4.76 ± 4.06) × 10^9^/L and (2.83 ± 0.96) × 10^9^/L; this result is consistent with the findings of Wu et al. that in the early stage of sepsis, peripheral blood WBC trend decreases at first and then increases. Hence, for postoperative patients with dynamic onitoring of WBC, if the changes show a downward trend, urosepsis should be considered rather than waiting for the WBC to rise significantly. It should be noticed that in the LPS 1000 group, the platelet count increases significantly and reaches (685.80 ± 150.52) × 10^9^/L at 1 hour after operation, which is much higher than that in the sham group, and the platelet level is maintained until 6 hours after the operation ((594.75 ± 240.02) × 10^9^/L). However, according to sepsis guideline, the lower the platelet count, the higher the SOFA score, that is, the more evidence for the diagnosis of sepsis. Thiery-Antier et al. also reported that decrease of platelet within 24 hours after the diagnosis of sepsis indicates a higher 28-day mortality rate [27]. Considering the changing trend of WBC in urosepsis, we give the hypothesis that in the early stage of urosepsis, the peripheral blood platelet count may increase first and then decrease and the increase of platelet count has a greater value in the early diagnosis of urosepsis.

In addition to platelet, serum histone H3 also increases significantly at 1 hour after operation. In the LPS 600 group, serum histone H3 reaches (5.71 ± 0.32) × 10^9^/L which is higher than that in the sham group and the gap grows over time. 6 hours after the operation, H3 level in the LPS 600 and LPS 1000 groups is (6.92 ± 0.55) × 10^9^/L and (7.45 ± 0.45) × 10^9^/L, respectively. ROC curve analysis finds that H3 can predict urosepsis with an AUC of 1.00. When setting 5.04 as the cut-off value by the Youden index, we find that serum H3 ≥ 5.04 has a sensitivity of 100% and specificity of 100% (Youden index: 1), which is higher than platelet and MMP-9. After analyzing ELISA data, we find that the serum H3 contents in the noninfected groups (control and sham group) and the LPS-treated groups have almost no crossover. 1 hour after the operation, serum H3 level in the noninfected groups is lower than 4.9 ng/mL while in the LPS-treated groups is all higher than 5.1 ng/mL. Thus, when using any concentration between 4.9 and 5.1 ng/mL as a critical threshold to distinguish infection, the extreme case of sensitivity and specificity of 100% occurs. This may due to insufficient sample size but we can still consider histone H3 as a potential biomarker for early diagnosis of urosepsis. Histone H3 as the main cytotoxic protein in the five subtypes of histone can directly damage endothelia cells, activate the inflammatory signaling pathway, and cause the mass release of inflammatory cytokines. H3 interacts with the phospholipid bimolecular layer of the cell membrane to promote the formation of channels and destroy the barrier structure of the cell membrane. As an important component of the neutrophil extracellular trap (NETs), histone is secreted by activated neutrophils when inflammation occurs, and Toll-like receptors-2/4 (TLR-2/4) triggered NF-*κ*B depended inflammatory signaling pathway which promotes the recruiment of WBCs in the microvasculature, thus mediating the occurrence of inflammation and tissue damage [13–15, 18, 19, 28]. This suggests that H3 plays an important role in the development of inflammatory process in the body. In addition to having great early diagnostic potential, antagonizing H3 may also become a viable treatment for urosepsis.

We find H3 levels in 1, 3, and 6 hours after the operation are significantly increased, but there is no significant change in peripheral blood neutrophils between groups after the operation (Tables 7–9). There may be two reasons behind the change: (1) When inflammation is induced, neutrophils are more efficiently active in H3 secretion, which occurs before the number of neutrophils rises. (2) Mass production of H3 in peripheral blood is derived from apoptotic or dead cells in the inflammatory process. Hence, uncovering the source of H3 in the early stage of urosepsis with massive blood intake still needs further study. Matrix metalloproteinases (MMP-9) and tissue inhibitor of metalloproteinase-1 (TIMP-1) are newly discovered inflammatory cytokines. Clinical trials have confirmed that the serum levels of MMP-9 and TIMP-1 increased significantly on the first day of sepsis occurrence, beginning to decrease on the third day, and the increase of concentration is especially evident in the serum of deceased patients [29, 30]. We find that TIMP-1 has no significant change in the early stage of urosepsis; MMP-9 increases significantly 1 hour after the operation but only in the LPS 1000 group. When the diagnostic point is 73.89 ng/mL, the diagnostic sensitivity is 60% and the specificity is 90%, which have certain diagnostic significance but are not as good as that of histone H3. Therefore, the diagnostic capacity of MMP-9 in the early stage of urosepsis is yet to be verified.

To sum up, ligating the ureter after an injection of 1000 *μ*g/kg LPS into the ureter of the rabbit can establish the animal model of urosepsis. On the basis of a realistic simulation of the pathogenesis of urosepsis, this method ensures a long enough survival time to collect clinical data and specimens. The increase of serum histone H3 can be detected within 1 hour of the infection with high diagnostic sensitivity and specificity of urosepsis as well, which is a sufficient biomarker for the early diagnosis of urosepsis. Furthermore, peripheral platelet count and serum MMP-9 concentration are also potential indexes. Whether these indexes can be used as biomarkers in clinical diagnosis needs to be further verified by clinical trials in the future.

## Figures and Tables

**Figure 1:** Changes of MAP postoperation. MAP of the LPS 600 group was significantly lower than the sham group (*P* = 0.048). MAP of the LPS 1000 group was significantly lower than the sham group (*P* < 0.001).

**Figure 2:** Changes of rectal temperature postoperation. Rectal temperature of the sham group significantly decreased compared with the control group (*P* = 0.002); temperature of the LPS 1000 group significantly decreased at 6 h postoperation compared with the sham group (*P* = 0.006).

**Figure 3:** Changes of leukocyte count postoperation. Leukocyte counts of the LPS 600 (*P* = 0.037) and the LPS 1000 group (*P* = 0.007) were significantly decreased at 3 h postoperation compared with the sham group; similar change was observed at 6 h postoperation in the 2 groups (*P* = 0.045 and *P* = 0.017).

**Figure 4:** Changes of platelet count postoperation. Platelet count of LPS 1000 was significantly increased at 1 h (*P* = 0.005), 3 h (*P* = 0.002), and 6 h (*P* = 0.041) postoperation compared with the sham group.

**Figure 5:** Changes of concentration of H3 postoperation. Concentration of H3 of the LPS 600 and the LPS 1000 groups significantly increased at 1 h (*P* = 0.001, *P* < 0.001), 3 h (*P* < 0.001 in both groups), and 6 h (*P* = 0.001, *P* < 0.001) postoperation.

**Figure 6:** Changes of MMP-9 postoperation. Concentration of MMP-9 of the LPS 1000 group significantly increased at 1 h (*P* < 0.001), 3 h (*P* = 0.003), and 6 h (*P* = 0.001) postoperation.

**Figure 7:** Postoperative 1 h ROC curve of indexes. All parameters above but MMP-9 (*P* = 0.174) had a diagnosis value (*P* < 0.05). AUC of H3, leukocyte, and platelet was 1.000, 0.810, and 0.950, respectively.

**Figure 8:** Postoperative 3 h ROC curve of indexes. All parameters above but MMP-9 (*P* = 0.112) had a diagnosis value (*P* < 0.05). AUC of H3, platelet, and leukocyte was 1.000, 0.920, and 0.911, respectively.

**Figure 9:** Postoperative 6 h ROC curve of indexes. All parameters above had a diagnosis value (*P* < 0.05). AUC of H3, leukocyte, platelet, and MMP-9 was 1.000, 0.852, 0.864, and 0.802, respectively.

**Figure 10:** Pathology of myocardial at 24 h postoperation (HE, 20x).

**Figure 11:** Pathology of alveoli at 24 h postoperation (HE, 20x).

**Figure 12:** Pathology of liver lobule at 24 h postoperation (HE, 20x).

**Figure 13:** Pathology of renal tubular at 24 h postoperation (HE, 20x).

**Table 1:** Comparison of vital signs among groups immediately after operation ($\bar{x}\pm s$).

Parameters	Groups				*F*	*P*	Multiple comparison	
	Control (*n* = 5)	Sham (*n* = 5)	LPS 600 (*n* = 5)	LPS 1000 (*n* = 5)			LSD test^a^	Dunnett *t*-test^b^
Cardiac rate (times/minute)	168.80 ± 71.89	223.60 ± 68.04	213.80 ± 51.89	155.40 ± 26.06	1.691	0.209	—	—
Respiratory rate (times/minute)	26.80 ± 10.18	28.00 ± 10.00	27.20 ± 10.52	37.40 ± 17.33	0.832	0.495	—	—
Rectal temperature (°C)	37.56 ± 0.86	35.18 ± 1.14	35.98 ± 0.93	36.06 ± 0.70	5.808	0.007^c^	0.001 0.189 0.150	-0.333 0.274
MAP (kPa)	7.91 ± 1.03	7.93 ± 1.29	7.96 ± 1.69	7.75 ± 0.78	0.029	0.993	—	—

^a^LSD test was between the control group vs. sham group, sham group vs. LPS 600 group, and sham group vs. LPS 1000 group, respectively, and same as what follows. ^b^Dunnett *t*-test was between the LPS 600 group vs. sham group and LPS 1000 group vs. sham group, and same as what follows. ^c^For rectal temperature, significant difference exists among groups (*P* < 0.01), which just comes from difference between the control group and sham group (*P* < 0.005).

**Table 2:** Comparison of vital signs among groups 1 h postoperation ($\bar{x}\pm s$).

Parameters	Groups				*F*	*P*	Multiple comparison	
	Control (*n* = 5)	Sham (*n* = 5)	LPS 600 (*n* = 5)	LPS 1000 (*n* = 5)			LSD test	Dunnett *t*-test
Cardiac rate (times/minute)	160.60 ± 52.86	224.80 ± 50.66	185.00 ± 55.11	175.00 ± 36.28	1.559	0.238	—	—
Respiratory rate (times/minute)	28.20 ± 5.81	36.60 ± 15.96	37.60 ± 28.43	39.00 ± 19.96	0.317	0.813	—	—
Rectal temperature (°C)	37.10 ± 0.91	35.40 ± 1.71	35.58 ± 0.69	35.90 ± 0.46	2.627	0.086	—	—
MAP (kPa)	8.86 ± 1.32	8.89 ± 0.70	7.74 ± 1.98	7.78 ± 1.60	0.949	0.440	—	—

No significant difference was found in parameters above.

**Table 3:** Comparison of vital signs among groups 3 h postoperation ($\bar{x}\pm s$).

Parameters	Groups				*F*	*P*	Multiple comparison	
	Control (*n* = 5)	Sham (*n* = 5)	LPS 600 (*n* = 5)	LPS 1000 (*n* = 5)			LSD test	Dunnett *t*-test
Cardiac rate (times/minute)	186.40 ± 92.09	223.30 ± 58.65	227.40 ± 45.48	163.00 ± 24.67	1.321	0.304	—	—
Respiratory rate (times/minute)	40.00 ± 9.49	46.60 ± 12.24	44.60 ± 31.99	55.25 ± 20.61	0.421	0.421	—	—
Rectal temperature (°C)	36.82 ± 0.54	35.12 ± 0.75	35.38 ± 0.97	35.35 ± 0.51	5.655	0.009^a^	0.002 0.580 0.644	-0.826 0.874
MAP (kPa)	9.71 ± 1.13	9.77 ± 0.71	8.12 ± 1.18	6.01 ± 1.13	12.405	<0.001^b^	0.932 0.025 <0.001	0.048 <0.001

^a^Significant difference of rectal temperature exists among groups (*P* < 0.01), which just comes from difference between the control group and sham group (*P* = 0.002 < 0.005). ^b^Significant difference of MAP exists among groups (*P* ≤ 0.001), which comes from difference between the LPS 600 group and sham group (*P* = 0.05) and between the LPS 1000 group and sham group (*P* < 0.001).

**Table 4:** Comparison of vital signs among groups 6 h postoperation ($\bar{x}\pm s$).

Parameters	Groups				*F*	*P*	Multiple comparison	
	Control (*n* = 5)	Sham (*n* = 5)	LPS 600 (*n* = 5)	LPS 1000 (*n* = 4)			LSD test	Dunnett *t*-test
Cardiac rate (times/minute)	221.40 ± 134.20	225.40 ± 128.19	223.80 ± 74.32	130.0 ± 11.80	0.863	0.482	—	—
Respiratory rate (times/minute)	53.60 ± 24.43	50.80 ± 14.04	45.00 ± 17.07	33.25 ± 15.78	1.039	0.404	—	—
Rectal temperature (°C)	37.74 ± 1.04	37.20 ± 0.60	35.12 ± 1.47	34.50 ± 1.71	7.372	0.003^a^	0.503 0.018 0.006	-0.052 0.020
MAP (kPa)	9.22 ± 0.89	9.25 ± 1.76	8.44 ± 1.48	8.00 ± 1.05	0.921	0.454	—	—

^a^Significant difference of rectal temperature exists among groups (*P* < 0.05), which just comes from difference between the LPS 1000 group and sham group (*P* = 0.002 < 0.005). ^b^Significant difference of MAP exists among groups (*P* ≤ 0.05).

**Table 5:** Comparison of vital signs among groups 12 h postoperation ($\bar{x}\pm s$).

Parameters	Groups				*F*	*P*	Multiple comparison	
	Control (*n* = 5)	Sham (*n* = 5)	LPS 600 (*n* = 5)	LPS 1000 (*n* = 4)			LSD test	Dunnett *t*-test
Cardiac rate (times/minute)	238.20 ± 88.65	220.80 ± 75.64	227.40 ± 86.39	143.00 ± 34.86	1.367	0.291	—	—
Respiratory rate (times/minute)	60.20 ± 18.74	54.40 ± 17.18	49.20 ± 19.97	49.00 ± 22.18	0.355	0.786	—	—
Rectal temperature (°C)	39.02 ± 0.62	38.34 ± 0.59	35.34 ± 2.40	34.93 ± 1.77	8.523	0.002^a^	0.495 0.008 0.005	-0.037 0.026
MAP (kPa)	9.68 ± 1.81	9.08 ± 1.29	7.48 ± 1.68	9.73 ± 1.00	2.334	0.115	—	—

^a^Significant difference of rectal temperature exists among groups (*P* < 0.005), which comes from difference between the LPS 600 group and sham group (*P* ≤ 0.05) and between the LPS 1000 group and sham group (*P* ≤ 0.05).

**Table 6:** Comparison of vital signs among groups 24 h postoperation ($\bar{x}\pm s$).

Parameters	Groups				*F*	*P*	Multiple comparison	
	Control (*n* = 5)	Sham (*n* = 5)	LPS 600 (*n* = 4)	LPS 1000 (*n* = 4)			LSD test	Dunnett *t*-test
Cardiac rate (times/minute)	256.80 ± 86.90	209.60 ± 64.90	176.75 ± 98.21	154.75 ± 50.91	1.491	0.260	—	—
Respiratory rate (times/minute)	58.00 ± 22.51	45.60 ± 11.93	42.00 ± 13.00	55.00 ± 13.71	0.982	0.429	—	—
Rectal temperature (°C)	38.84 ± 0.57	39.02 ± 0.55	35.48 ± 3.56	37.20 ± 2.20	3.046	0.064	—	—
MAP (kPa)	9.71 ± 1.49	8.74 ± 1.05	6.09 ± 3.50	8.57 ± 1.42	2.453	0.110	—	—

No significant difference was found in parameters above.

**Table 7:** Comparison of routine blood and CRP among groups 1 h postoperation ($\bar{x}\pm s$).

Parameters	Groups				*F*	*P*	Multiple comparison	
	Control (*n* = 5)	Sham (*n* = 5)	LPS 600 (*n* = 5)	LPS 1000 (*n* = 5)			LSD test	Dunnett *t*-test
Erythrocyte count (10^12^/L)	6.39 ± 0.71	6.84 ± 1.17	6.68 ± 0.83	6.66 ± 0.53	0.246	0.863	—	—
Leukocyte count (10^9^/L)	6.36 ± 1.31	6.60 ± 4.18	5.90 ± 7.24	2.30 ± 1.06	1.117	0.372	—	—
Neutrophil count (10^9^/L)	2.32 ± 1.19	2.10 ± 1.89	1.61 ± 2.82	0.26 ± 0.13	1.317	0.304	—	—
Hemoglobin (g/L)	129.80 ± 15.07	135.20 ± 14.10	139.40 ± 23.78	123.80 ± 11.08	0.820	0.501	—	—
Platelet count (10^9^/L)	180.00 ± 70.06	257.20 ± 136.34	456.80 ± 231.59	685.80 ± 150.52	10.340	0.001^a^	0.451 0.053 0.001	0.153 0.005
CRP (mg/L)	75.49 ± 1.56	75.63 ± 2.52	77.98 ± 4.57	78.20 ± 0.86	1.413	0.276	—	—

^a^Significant difference of platelet count exists among groups (*P* < 0.005), which just comes from difference between the LPS 1000 group and sham group (*P* ≤ 0.01).

**Table 8:** Comparison of routine blood and CRP among groups 3 h postoperation ($\bar{x}\pm s$).

Parameters	Groups				*F*	*P*	Multiple comparison	
	Control (*n* = 5)	Sham (*n* = 5)	LPS 600 (*n* = 5)	LPS 1000 (*n* = 5)			LSD test	Dunnett *t*-test
Erythrocyte count (10^12^/L)	6.00 ± 0.59	6.78 ± 1.18	7.21 ± 1.07	6.39 ± 0.99	1.383	0.284	—	—
Leukocyte count (10^9^/L)	10.84 ± 2.71	9.84 ± 3.86	3.86 ± 4.74	1.74 ± 0.40	8.847	0.001^a^	0.643 0.012 0.002	0.037 0.007
Neutrophil count (10^9^/L)	4.10 ± 3.54	2.26 ± 2.48	0.90 ± 1.03	0.32 ± 0.04	2.858	0.07	—	—
Hemoglobin (g/L)	121.20 ± 9.93	131.40 ± 16.59	136.20 ± 23.49	117.40 ± 20.96	1.118	0.371	—	—
Platelet count (10^9^/L)	251.60 ± 74.59	187.80 ± 108.62	402.80 ± 171.26	633.60 ± 206.74	8.779	0.001^b^	0.510 0.037 <0.001	0.113 0.002
CRP (mg/L)	74.80 ± 1.26	75.49 ± 3.23	77.64 ± 2.96	77.67 ± 1.23	1.958	0.161	—	—

^a^Significant difference of leukocyte count exists among groups (*P* = 0.001), which comes from difference between the LPS 600 group and sham group (*P* ≤ 0.05) and between the LPS 1000 group and sham group (*P* < 0.01). ^b^Significant difference of platelet count exists among groups (*P* = 0.001), which just comes from difference between the LPS 1000 group and sham group (*P* ≤ 0.005).

**Table 9:** Comparison of routine blood and CRP among groups 6 h postoperation ($\bar{x}\pm s$).

Parameters	Groups				*F*	*P*	Multiple comparison	
	Control (*n* = 5)	Sham (*n* = 5)	LPS 600 (*n* = 5)	LPS 1000 (*n* = 4)			LSD test	Dunnett *t*-test
Erythrocyte count (10^12^/L)	5.49 ± 1.78	5.86 ± 0.86	7.11 ± 1.25	5.64 ± 1.37	1.464	0.264	—	—
Leukocyte count (10^9^/L)	10.26 ± 5.42	11.36 ± 5.24	4.76 ± 4.06	2.83 ± 0.96	4.013	0.028^a^	0.701 0.033 0.012	0.045 0.017
Neutrophil count (10^9^/L)	4.76±4.00	4.42±3.58	1.18±0.90	1.08±0.51	18.971	0.11	—	—
Hemoglobin (g/L)	108.80 ± 26.41	110.80 ± 14.96	138.20 ± 25.17	105.75 ± 30.45	1.819	0.187	—	—
Platelet count (10^9^/L)	206.00 ± 92.80	234.20 ± 128.75	379.40 ± 231.25	594.75 ± 240.02	4.237	0.023^b^	0.808 0.222 0.009	0.449 0.041
CRP (mg/L)	75.86 ± 1.35	76.75 ± 2.01	77.64 ± 2.63	78.08 ± 0.79	1.108	0.379	—	—

^a^Significant difference of leukocyte count exists among groups (*P* = 0.028), which comes from difference between the LPS 600 group and sham group (*P* < 0.05) and between the LPS 1000 group and sham group (*P* < 0.05). ^b^Significant difference of platelet count exists among groups (*P* = 0.023), which just comes from difference between the LPS 1000 group and sham group (*P* < 0.005).

**Table 10:** Comparison of results of ELISA among groups 3 h postoperation ($\bar{x}\pm s$).

Parameters	Groups				*F*	*P*	Multiple comparison	
	Control (*n* = 5)	Sham (*n* = 5)	LPS 600 (*n* = 5)	LPS 1000 (*n* = 5)			LSD test	Dunnett *t*-test
PCT (pg/mL)	10.72 ± 2.13	13.98 ± 1.29	11.99 ± 2.68	11.21 ± 1.46	2.653	0.084	—	—
Histone H3 (ng/mL)	4.10 ± 0.49	4.13 ± 0.42	6.04 ± 0.21	6.49 ± 0.38	51.975	<0.001^a^	0.880 <0.001 <0.001	<0.001 <0.001
Histone H4 (ng/mL)	2.24 ± 0.26	2.49 ± 0.25	3.19 ± 0.24	3.46 ± 0.31	23.052	<0.001^b^	0.159 0.001 <0.001	0.003 <0.001
MMP-9 (ng/mL)	51.38 ± 3.94	59.11 ± 23.57	47.88 ± 20.41	136.10 ± 41.61	12.925	<0.001^c^	0.646 0.506 <0.001	0.783 0.003
TIMP-1 (ng/mL)	70.06 ± 12.93	82.10 ± 28.99	67.54 ± 15.39	52.93 ± 8.10	2.190	0.129	—	—

^a^Significant difference of concentration of H3 exists among groups (*P* < 0.001), which comes from difference between the LPS 600 group and sham group (*P* < 0.001) and between the LPS 1000 group and sham group (*P* < 0.001). ^b^Significant difference of concentration of H4 exists among groups (*P* < 0.001), which comes from difference between the LPS 600 group and sham group (*P* < 0.005) and between the LPS 1000 group and sham group (*P* < 0.001). ^c^Significant difference of concentration of MMP-9 exists among groups (*P* < 0.001), which just comes from difference between the LPS 1000 group and sham group (*P* < 0.005).

**Table 11:** Comparison of results of ELISA among groups 6 h postoperation ($\bar{x}\pm s$).

Parameters	Groups				*F*	*P*	Multiple comparison	
	Control (*n* = 5)	Sham (*n* = 5)	LPS 600 (*n* = 5)	LPS 1000 (*n* = 4)			LSD test	Dunnett *t*-test
PCT (pg/mL)	14.37 ± 5.55	15.08 ± 5.19	11.94 ± 1.61	10.62 ± 3.39	1.093	0.384	—	—
Histone H3 (ng/mL)	4.57 ± 0.42	4.32 ± 0.39	6.92 ± 0.55	7.45 ± 0.45	57.107	<0.001^a^	0.384 <0.001 <0.001	0.001 <0.001
Histone H4 (ng/mL)	2.49 ± 0.19	2.59 ± 0.18	3.74 ± 0.30	3.68 ± 0.18	44.475	<0.001^b^	0.501 <0.001 <0.001	<0.001 <0.001
MMP-9 (ng/mL)	64.10 ± 25.71	48.92 ± 14.78	63.83 ± 25.53	111.55 ± 12.21	7.463	0.003^c^	0.290 0.271 <0.001	0.387 0.001
TIMP-1 (ng/mL)	87.59 ± 24.59	80.64 ± 26.89	79.11 ± 18.89	49.54 ± 11.52	2.479	0.104	—	—

^a^Significant difference of concentration of H3 exists among groups (*P* < 0.001), which comes from difference between the LPS 600 group and sham group (*P* < 0.001) and between the LPS 1000 group and sham group (*P* < 0.001). ^b^Significant difference of concentration of H4 exists among groups (*P* < 0.001), which comes from difference between the LPS 600 group and sham group (*P* < 0.05) and between the LPS 1000 group and sham group (*P* < 0.001). ^c^Significant difference of concentration of MMP-9 exists among groups (*P* < 0.001), which just comes from difference between the LPS 1000 group and sham group (*P* < 0.005).

**Table 12:** Comparison of results of ELISA among groups 1 h postoperation ($\bar{x}\pm s$).

Parameters	Groups				*F*	*P*	Multiple comparison	
	Control (*n* = 5)	Sham (*n* = 5)	LPS 600 (*n* = 5)	LPS 1000 (*n* = 5)			LSD test	Dunnett *t*-test
PCT (pg/mL)	9.46 ± 2.09	15.56 ± 9.81	11.40 ± 1.67	12.59 ± 2.79	1.176	0.350	—	—
Histone H3 (ng/mL)	3.89 ± 0.50	4.18 ± 0.60	5.71 ± 0.32	6.22 ± 0.57	25.031	<0.001^a^	0.385 <0.001 <0.001	0.001 <0.001
Histone H4 (ng/mL)	2.32 ± 0.18	2.39 ± 0.30	2.89 ± 0.29	3.32 ± 0.26	15.747	<0.001^b^	0.676 0.008 <0.001	0.030 <0.001
MMP-9 (ng/mL)	57.71 ± 19.22	42.79 ± 9.53	47.00 ± 20.91	120.18 ± 18.46	20.997	<0.001^c^	0.199 0.710 <0.001	0.896 <0.001
TIMP-1 (ng/mL)	76.14 ± 15.07	80.36 ± 20.65	62.24 ± 26.40	50.91 ± 6.18	2.606	0.088	—	—

^a^Significant difference of concentration of H3 exists among groups (*P* < 0.001), which comes from difference between the LPS 600 group and sham group (*P* < 0.005) and between the LPS 1000 group and sham group (*P* < 0.001). ^b^Significant difference of concentration of H4 exists among groups (*P* < 0.001), which comes from difference between the LPS 600 group and sham group (*P* < 0.05) and between the LPS 1000 group and sham group (*P* < 0.001). ^c^Significant difference of concentration of MMP-9 exists among groups (*P* < 0.001), which just comes from difference between the LPS 1000 group and sham group (*P* < 0.001).

**Table 13:** Comparison of diagnostic capability of parameters at 1 h postoperation.

Parameter	Cut-off	AUC	Standard error	95% CI	*P* ^a^	Sensibility (%)	Specificity (%)
Leukocyte count (10^9^/L)	3.8	0.810	0.106	0.602-1.000	0.019	80.0	80.0
Platelet count (10^9^/L)	305.5	0.950	0.045	0.862-1.000	0.001	90.0	90.0
H3 (ng/mL)	5.04	1.000	<0.001	1.000-1.000	<0.001	100.0^b^	100.0^b^
MMP-9 (ng/mL)	73.89	0.680	0.131	0.424-0.936	0.174	60.0	90.0

**Table 14:** Comparison of diagnostic capability of parameters at 3 h postoperation.

Parameter	Cut-off	AUC	Standard error	95% CI	*P* ^a^	Sensibility (%)	Specificity (%)
Leukocyte count (10^9^/L)	3.8	0.920	0.078	0.767-1.000	0.001	90.0	100.0
Platelet count (10^9^/L)	305.5	0.920	0.065	0.792-1.000	0.001	90.0	90.0
H3 (ng/mL)	5.04	1.000	<0.001	1.000-1.000	<0.001	100.0^b^	100.0^b^
MMP-9 (ng/mL)	73.89	0.710	0.125	0.464-0.956	0.112	60.0	90.0

**Table 15:** Comparison of diagnostic capability of parameters at 6 h postoperation.

Parameter	Cut-off	AUC	Standard error	95% CI	*P* ^a^	Sensibility (%)	Specificity (%)
Leukocyte count (10^9^/L)	6.4	0.867	0.089	0.693-1.000	0.007	88.9	80.0
Platelet count (10^9^/L)	345.5	0.856	0.100	0.659-1.000	0.009	90.0	90.0
H3 (ng/mL)	5.6	1.000	<0.001	1.000-1.000	<0.001	100.0^b^	100.0^b^
MMP-9 (ng/mL)	94.35	0.822	0.097	0.633-1.000	0.018	55.6	100.0

^a^ *P* < 0.05 means the parameter had a diagnosis value. ^b^For data of histone H3 and H4, the minimum in the experimental group was greater than maximum in the sham and control groups, so the sensibility and specificity were 100%.

## Data Availability

All the data would be provided if required.

## Supplementary Materials

Supplementary Materials Supplemental Figure S1: postoperative changes of heart rate. Supplemental Figure S2: postoperative changes of respiratory rate. Supplemental Figure S3: postoperative changes of CRP level. Supplemental Figure S4: postoperative changes of PCT level. Supplemental Figure S5: postoperative changes of TIMP-1 level.
